# Silencing lncRNA XIST exhibits antiproliferative and proapoptotic effects on gastric cancer cells by up-regulating microRNA-132 and down-regulating PXN

This article has been retracted.

**DOI:** 10.18632/aging.103635

**Published:** 2020-11-05

**Authors:** Ping Li, Liuhua Wang, Pengfei Li, Fangyong Hu, Yi Cao, Dong Tang, Gang Ye, Hongbo Li, Daorong Wang

**Affiliations:** 1 Department of General Surgery, Huaian Tumor Hospital, Huaian Hospital of Huaian City, Huaian, 223200, P.R. China; 2 Department of Experimental Surgery-Cancer Metastasis, Medical Faculty Mannheim, Ruprecht Karls University, Mannheim 68167, Germany; 3 Department of General Surgery, Northern Jiangsu Province Hospital, Clinical Medical College, Institute of General Surgery - Yangzhou, Yangzhou University, Yangzhou 225000, P.R. China; 4 Department of General Surgery, Jiangdu People's Hospital of Yangzhou, Yangzhou 225200, P.R. China

**Keywords:** gastric cancer, long non-coding RNA XIST, MicroRNA-132, paxillin, proliferation

## Abstract

The present study aims to elucidate the potential therapeutic role of lncRNA XIST in gastric cancer through regulation of microRNA-132 (miR-132) and paxillin (PXN) expression. The study employed 65 gastric cancer tissue specimens and SGC7901 cell lines. Our results demonstrated that expression of lncRNA XIST and PXN was significantly elevated while the expression of miR-132 was significantly reduced in gastric cancer tissues. Dual-luciferase, RNA pull-down and RIP assays demonstrated that lncRNA XIST up-regulated the PXN expression by competitively binding to miR-132. Moreover, silencing of lncRNA XIST and up-regulation of miR-132 could suppress tumor formation ability, cell proliferation and migration, but enhanced apoptosis in gastric cancer. However, the overexpression of PXN achieved the opposite tumor-promotive effect. Meanwhile, rescue experiments suggested that silencing of lncRNA XIST could reverse the tumor-promotive effect exerted by either miR-132 inhibitor or PXN. Taken together, the present study demonstrates lncRNA XIST as a novel oncogenic lncRNA in gastric cancer, highlighting its therapeutic role in this disease.

## INTRODUCTION

Gastric cancer is a common malignancy and one of the leading cancer-related death causes across the globe. Infection with *Helicobacter pylori* is known as the most dominant risk factor for gastric cancer [1]. The average survival rate of gastric cancer patients post diagnosis remains depressingly poor at merely 8 - 10 months, despite the usage of effective chemotherapeutic drugs such as irinotecan, taxanes, fluoropyrimidine and platinum base [2]. Poor prognosis in patients with malignancy still occurs, in large part, due to the difficulty of early detection; GC is often not diagnosed until it evolves to x stage [3]. Also, the fatality rate of gastric cancer was as high as 75%. Currently, prevention of gastric cancer is performed by radiological or endoscopic screening methods with limiting success [4]. The long non-coding RNA (lncRNA) is implicated in cell migration and lymph node metastasis of gastric cancer cells [5]. MicroRNAs (miRs) are associated with multiple cellular activities, including immune function, metabolism, cell apoptosis and growth of gastric cancer [6].

Paxillin (PXN) is known as a focal adhesion adapter protein with multiple functions in a variety of domains, which exerts a vital influence in focal adhesion, tumor progression and migration, barrier dysfunction of endothelial cells, inflammatory reaction and oxidative stress [7]. Meanwhile, the aberrant expression of PXN is often found in human cancer progression, and the correlation between PXN and the invasiveness of gastric cancer cell line AGS has also been reported [8]. The lncRNA X-inactive specific transcript (XIST) is encoded by the X chromosome and functions in human cell gene maintenance, proliferation and differentiation [9]. Previous findings revealed that miR-137-induced knockdown of PXN can accelerate the metastasis and development of colorectal cancer [10]. miR-132 might serve as a promising prognostic factor in gastric cancer by affecting angiogenesis, inflammation and the neuro-development [11]. We aim to test the effect of lncRNA XIST on gastric cancer since both lncRNA XIST and PXN were predicted to bind to miR-132 according to the computer-based lncRNA-miR-mRNA interaction analysis. This study will provide a more solid understanding of the underlying molecular mechanisms that govern the lncRNA XIST, miR-132 and PXN interactions in tumor formation ability, cell proliferation, migration and apoptosis of gastric cancer and hopefully lead to better diagnostic and therapeutic tools.

## RESULTS

### LncRNA XIST is highly expressed in gastric cancer tissues

The expression of lncRNA XIST in gastric cancer tissues and adjacent normal tissues was determined first using RT-qPCR, which found higher expression of lncRNA XIST in gastric cancer tissues (*p* < 0.001) (Figure 1A). Meanwhile, among our cohort of 65 gastric cancer tissue samples, the relative expression of lncRNA XIST was significantly lower in non-metastatic tissues (n = 20) than in metastatic tissues (n = 45) (*p* = 0.001) (Figure 1B). Relative to the normal gastric epithelial cell line GSE-1, all gastric cancer cell lines exhibited an elevated lncRNA XIST expression (Figure 1C), with the highest lncRNA XIST expression determined in SGC7901 cells. Thus, SGC7901 cells were selected for the following functional experiments. FISH (Figure 1D) illustrated the expression of lncRNA XIST in the cytoplasm. Taken together, these results unraveled elevated expression of lncRNA XIST in gastric cancer tissues.

**Figure 1:** **LncRNA XIST is highly expressed in gastric cancer tissues and cell lines.** (**A**) Relative expression of lncRNA XIST in gastric cancer tissues (n = 65) and the adjacent normal tissues determined by RT-qPCR; *, *p* < 0.05 compared with adjacent normal tissues; (**B**) Relative expression of lncRNA XIST in gastric cancer tissues from patients with metastasis (n = 45) and without metastasis (n = 20) determined by RT-qPCR; *, *p* < 0.05 compared with gastric cancer tissues from patients without metastasis; (**C**) Relative expression of lncRNA XIST in different gastric cancer cell lines; *, *p* < 0.05 compared with the normal cells; #, *p* < 0.05 compared with the SGC7901 cells; (**D**) the representative images of localization of lncRNA XIST merged with DAPI wherein red signal represented lncRNA XIST and blue signal represented cell nucleus (× 200). All measurement data and statistical results were expressed as mean ± standard deviation. Comparisons between two groups were analyzed by *t*-test, while comparisons among multiple groups were analyzed using one-way ANOVA. The experiment was repeated 3 times.

### Knockdown of lncRNA XIST retards tumor formation ability, cell proliferation and migration, and induces apoptosis in gastric cancer cells

As stated above, the gastric cancer cell line SGC7901 was selected to evaluate the effects of lncRNA XIST on the biological functions of gastric cancer cells by conducting knockdown experiments. We successfully knocked down lncRNA XIST in cells transfected with si-XIST-1 and si-XIST-2 as shown by its lowered expression (Figure 2A).

**Figure 2:** **Inhibition of LncRNA XIST restrains tumor formation ability, cell proliferation and migration and enhances apoptosis in gastric cancer.** The SGC7901 cells were transfected with siRNAs targeting XIST, namely, si-XIST-1 and si-XIST-2. (**A**) The expression of lncRNA XIST determined by RT-qPCR; (**B**) Cell proliferation ability assessed by EdU assay (× 400); (**C**) Cell migration ability evaluated by scratch test (× 40); (**D**) Cell apoptosis ability evaluated by flow cytometry; (**E**) The effect of lncRNA XIST on tumor formation in nude mice injected with the stably transfected SGC7901 cells. All measurement data and statistical results were expressed as mean ± standard deviation; *, *p* < 0.05 compared with cells transfected with si-NC or the mice injected with si-NC-transfected cells; comparisons were conducted using one-way ANOVA. The experiment was repeated 3 times.

Next, EdU assay, scratch test, Transwell assay and flow cytometry were performed respectively to assess cell proliferation (Figure 2B), migration (Figure 2C) and apoptosis (Figure 2D). Two siRNAs for lncRNA XIST reduced SGC7901 cell proliferation and migration abilities but induced cell apoptosis rate (*p* < 0.05). No notable difference was found between SGC7901 cells introduced with si-XIST-1 and si-XIST-2. Tumor xenografts in nude mice (Figure 2E) showed that tumor volume was gradually increased over time. The tumor volume and weight in mice injected with the SGC7901 cells stably transfected with si-XIST-1 and si-XIST-2 at the same point were significantly decreased (*p* < 0.05), while no obvious differences were found between the mice injected with SGC7901 cells stably transfected with si-XIST-1 and si-XIST-2. Thus, depleting lncRNA XIST expression could suppress tumor formation ability, cell proliferation and migration and, promote cell apoptosis in gastric cancer.

### LncRNA XIST binds to miR-132 to affect gastric cancer cell progression

The bioinformatics online prediction predicted the binding region between lncRNA XIST and miR-132 (Figure 3A). Next, we verified this binding relationship using a dual luciferase reporter gene assay (Figure 3B). The luciferase activity in the miR-132 binding region with WT-lncRNA XIST was inhibited by miR-132 mimic, while that of MUT-lncRNA XIST was escaped from inhibition, suggesting that miR-132 could specifically bind to the lncRNA XIST. Results of the RIP assay (Figure 3C) demonstrated that when compared with IgG, Ago2 combined with lncRNA XIST and miR-132 was significantly increased (*p* < 0.05), thus showing that lncRNA XIST and miR-132 could bind to Ago2 protein. The results of the RNA pull-down assay (Figure 3D) suggested that the expression of WT-miR-132 binding to Ago protein was markedly increased when compared with MUT-miR-132 (*p* < 0.05), indicating that the direct binding relationship between miR-132 and lncRNA XIST was valid.

**Figure 3:** **MiR-132 specifically binds to lncRNA XIST and its overexpression restrains tumor formation ability, cell proliferation and migration while promoting apoptosis in gastric cancer.** (**A**) Binding region between miR-132 and lncRNA XIST; (**B**) Relative luciferase activity of miR-132 and lncRNA XIST; (**C**) Binding of lncRNA XIST to miR-132 and Ago2 detected by RIP assay; (**D**) RNA pull-down assay suggested binding relationship between lncRNA XIST and miR-132; (**E**) Relative expression of miR-132 in gastric cancer tissues (n = 65) and the adjacent normal tissues determined by RT-qPCR; *, *p* < 0.05 compared with adjacent normal tissues; (**F**) Relative expression of miR-132 in gastric cancer tissues from patients with metastasis (n = 45) and without metastasis (n = 20) determined by RT-qPCR; *, *p* < 0.05 compared with gastric cancer tissues from patients without metastasis; In the panels (**G**–**I**) SGC7901 cells were transfected with miR-132 mimic or inhibitor or co-transfected with miR-132 inhibitor and si-XIST. (**G**) Cell proliferation ability evaluated by EdU assay (× 400); (**H**) Cell migration ability assessed by scratch test (× 40); (**I**) Cell apoptosis ability in each group detected by flow cytometry; (**J**) The effect of miR-132 and lncRNA XIST on tumor formation in nude mice injected with the stably transfected SGC7901 cells. All measurement data and statistical results were expressed as mean ± standard deviation. A value of *p* < 0.05 was considered as statistically significant and a value of *p* < 0.001 was considered statistically highly significant; *, *p* < 0.05 compared with the NC group; comparisons between two groups were analyzed by *t*-test, while comparison among multiple groups were analyzed using one-way ANOVA. The experiment was repeated 3 times.

By RT-qPCR determination, miR-132 expression was reduced in gastric cancer tissues as compared to matched non-tumor tissues (*p* < 0.05) (Figure 3E). Furthermore, miR-132 expression was relatively higher in the gastric cancer tissues from patients without metastasis (n = 20) than in patients with metastasis (n = 45) (Figure 3F). Next, SGC7901 cells were transfected with miR-132 mimic or inhibitor or co-transfected with miR-132 inhibitor and si-XIST. The cell proliferation (Figure 3G), migration (Figure 3H) and apoptosis (Figure 3I) were then detected by EdU assay, scratch test, Transwell assay and flow cytometry, respectively. Results showed that the transfection with the miR-132 mimic contributed to reduced cell viability, migration ability and enhanced cell apoptosis (*p* < 0.05). On the other hand, transfection with miR-132 inhibitor resulted in significant elevation in cell viability, migration ability and a decrease in cell apoptosis rate (*p* < 0.05). In contrast with SGC7901 cells transfected with miR-132 inhibitor, those co-transfected with miR-132 inhibitor and si-XIST displayed decreased viability, migration ability and an enhanced apoptosis rate (*p* < 0.01).

Finally, a tumor xenograft model in nude mice was utilized to assess tumor formation ability of gastric cancer cells. Results displayed in Figure 3I showed that over time, tumor volume was significantly increased (*p* < 0.05). In contrast, the tumor volume and weight of mice injected with the SGC7901 cells stably transfected with miR-132 mimic at the same point was significantly decreased while those injected with the SGC7901 cells stably transfected with miR-132 inhibitor was significantly increased (*p* < 0.05). Moreover, the enhanced tumor growth by inhibition of miR-132 was inhibited by coinstantaneous lncRNA XIST silencing. Taken together, the overexpression of miR-132 could suppress tumor formation and cell proliferation while promoting apoptosis in gastric cancer while lncRNA XIST silencing could reverse the tumor-promotive effects of miR-132 inhibition on gastric cancer.

### LncRNA XIST binds to miR-132 and regulates its target gene PXN

The putative binding site between miR-132 and PXN was predicted by the bioinformatics online prediction and verified using a dual luciferase reporter gene assay. Result from bioinformatics online prediction (Figure 4A) revealed an existing binding site between miR-132 and 3’UTR region of PXN, suggesting that PXN was a target gene of miR-132. The dual-luciferase reporter gene assay (Figure 4B) demonstrated that the luciferase activity of WT-PXN 3’UTR was restrained by miR-132 (*p* < 0.05), while that of MUT-PXN 3’UTR was not affected (*p* > 0.05), indicating that miR-132 could specifically bind to PXN 3’UTR and down-regulate its expression after transcription.

**Figure 4:** **LncRNA XIST competitively binds to miR-132 and modulates PXN.** (**A**) Binding region between miR-132 and PXN; (**B**) Relative luciferase activity between miR-132 and PXN; (**C**) Protein bands of PXN measured by western blot assay; (**D**) PXN protein expression in the SGC7901 cells transfected with miR-132 mimic or inhibitor or co-transfected with miR-132 inhibitor and si-XIST. All measurement data and statistical results were expressed as mean ± standard deviation; *, *p* < 0.05 compared with the NC group. Comparisons between two groups were analyzed by *t*-test, while comparison among multiple groups were analyzed using one-way ANOVA. The experiment was repeated 3 times.

Next, the protein expression of PXN was determined by Western blot analysis. As depicted in Figure 4C, 4D, PXN protein expression was significantly reduced in cells transfected with miR-132 mimic, and was significantly increased in those transfected with miR-132 inhibitor (*p* < 0.05). In addition, the increase in PXN protein expression caused by miR-132 inhibitor was counteracted by si-XIST (*p* < 0.05). These results demonstrated that lncRNA XIST could competitively bind to miR-132 and upregulate PXN.

### LncRNA XIST upregulates PXN to elevate gastric cancer progression and tumorigenesis *in vitro* and *in vivo*

As determined by RT-qPCR, PXN expression was significantly higher in gastric cancer tissues than in matched non-tumor tissues (*p* < 0.05) (Figure 5A), and the PXN expression in the gastric cancer tissues from patients without metastasis (n = 20) was increased compared to those from patients with metastasis (n = 45) (Figure 5B). We overexpressed PXN cells in SGC7901 to analyze the influence of PXN on biological functions of gastric cancer cells. Successful transfection was indicated by results showing that the expression of PXN in the oe-PXN-1 and oe-PXN-2 groups was markedly increased when compared with the oe-NC group (Figure 5C).

**Figure 5:** **PXN enhances tumor formation ability, cell proliferation and metastasis, but suppresses cell apoptosis in gastric cancer.** (**A**) Relative expression of PXN in gastric cancer tissues (n = 65) and the adjacent normal tissues determined by RT-qPCR; *, *p* < 0.05 compared with adjacent normal tissues; (**B**) Relative expression of PXN in gastric cancer tissues from patients with metastasis (n = 45) and without metastasis (n = 20) determined by RT-qPCR; *, *p* < 0.05 compared with gastric cancer tissues from patients without metastasis; In the panels (**C**–**F**), SGC7901 cells were transfected with oe-PXN or co-transfected with oe-PXN and si-XIST. (**C**) The mRNA expression of PXN detected by RT-qPCR; (**D**) Cell proliferation ability in each group detected by EdU assay (× 400); (**E**) Cell migration ability detected by scratch test (× 40); (**F**) Cell apoptosis ability detected by flow cytometry; (**G**) The effect of PXN and lncRNA XIST on tumor formation in nude mice injected with the stably transfected SGC7901 cells. All measurement data and statistical results were expressed as mean ± standard deviation. *, *p* < 0.05 compared with cells transfected with oe-NC or the mice injected with the oe-NC-transfected cells. Comparisons among multiple groups were analyzed using one-way ANOVA. The experiment was repeated 3 times.

Next, cell proliferation (Figure 5D), migration (Figure 5E), apoptosis (Figure 5F) and tumor formation ability (Figure 5G) were measured by EdU assay, scratch test, Transwell assay, flow cytometry, and *in vivo* experiments, respectively. Results demonstrated that overexpression of PXN led to significant increased cell viability, migration ability as well as tumorigenicity of SGC7901 cells but reduction in cell apoptosis rate (*p* < 0.05). In our tumor model, tumor volume was gradually increased over time. Thus, PXN overexpression could promote tumor formation ability, cell proliferation and migration but inhibit cell apoptosis in gastric cancer. However, the stimulative effects of PXN on the cell growth, migration and tumorigenicity and its inhibitory effect on cell apoptosis were neutralized by lncRNA XIST silencing.

## DISCUSSION

Gastric cancer is a leading cause of tumor-induced death worldwide, accompanied by high occurrence and mortality rates. This may be caused by insufficient diagnoses at early stages coupled with inefficient therapeutic treatments at advanced stages [12, 13]. Currently, patients with gastric cancer at an advanced stage, can undergo chemotherapy, bypass surgery or palliative resection and gastrectomy, however, this still results in unsatisfactory prognosis [14]. Accumulating research contributes to advancement in carcinogenesis and anti-cancer drug development [15–17]. A recent study has reported the potential regulatory roles of miRs and lncRNAs in tumor formation and development of gastric cancer [18]. Our study revealed that silencing of the lncRNA XIST could inhibit gastric cancer cell proliferation and migration, while promoting apoptosis, all this being achieved through up-regulating miR-132 and consequently, reducing PXN expression.

Our initial findings revealed that lncRNA XIST and PXN were highly expressed, while miR-132 was poorly expressed in gastric cancer. A previous study has shown that lncRNA XIST can act as an oncogenic lncRNA with higher expression in hepatocellular carcinoma, non-small cell lung cancer as well as gastric cancer, which was in line with our finding [19–21]. The high expression of lncRNA urothelial carcinoma associated 1 (UCA1) is detected in gastric cells and tissues, which is similar to our study [22]. In addition, PXN expression is increased in gastric adenoma compared to adjacent non-cancerous mucosa, and this abnormal expression is correlated with gastric cancer differentiation, metastasis and proliferation [23]. Furthermore, poor miR-132-3p expression has been detected in gastric cancer, which facilitates gastric cancer cell growth and migration [24].

In addition, our target prediction program in conjunction with a dual-luciferase activity assay, verified that lncRNA XIST bound to miR-132, causing reduced XIST and upregulated miR-132, hence suppressing gastric cancer cell proliferation and migration that induced by PXN overexpression. An increase in PXN expression facilitates tumor invasion and metastasis in gastric cancer, yet miR-212 can serve as an anti-oncogene to suppress gastric cancer metastasis by lowering PXN [25]. In support of this, lncRNA XIST is known to sponge miR-101 and thus affects the progression of gastric cancer, which may constitute a preventive therapeutic method for treating gastric cancer [26]. Meanwhile, lncRNA XIST is linked to colorectal cancer cell proliferation through knockdown of miR-132-3p [27]. Moreover, lncRNA XIST also participates in the viability of non-small cell lung cancer cells *via* sponging miR-137 and regulating PXN expression [9]. Additionally, lncRNA nuclear-enriched abundant transcript 1 (NEAT1) has been shown to be involved in gastric cancer cell migration and proliferation *via* up-regulating miR-17 [28].

In addition, our findings provide evidence that silencing of lncRNA XIST restrained tumor formation ability, cell proliferation and migration, yet promoted apoptosis in gastric cancer by elevating miR-132 and inhibiting PXN. In accordance with our result, a previous study has also revealed that knockdown of lncRNA XIST contributes to the depressed human glioblastoma stem cell migration and proliferation as well as enhances apoptosis through up-regulation of miR-152 [29]. More importantly, inhibition of lncRNA XIST contributes to suppressed proliferation of gastric cancer cells by sponging miR-497 and restraining metastasis-associated in colon cancer 1 (MACC1) [21]. Also, silencing of lncRNA XIST has also been found to decrease cell metastasis, and growth in bladder cancer through interaction with miR-124 and androgen receptor [30]. Additionally, the silenced lncRNA CCAT2 has been reported to restrain cell migration and proliferation in gastric cancer [31].

In conclusion, the key findings of the study demonstrated that depletion of lncRNA XIST inhibited gastric cancer progression through elevation of miR-132 and inhibition of PXN. These findings may be instrumental for the development of therapeutic targets and clinical management of gastric cancer. However, further in-depth studies involving lncRNA XIST, miR-132 and PXN in clinical samples with a large-scale sample size are required for a better understanding.

## MATERIALS AND METHODS

### Ethics statement

The protocols of the present study were approved by the Institutional Review Board of Northern Jiangsu Province Hospital, Clinical Medical College, Institute of General Surgery - Yangzhou, Yangzhou University. Written informed consents were signed by all participating patients. The study was carried out in strict accordance with the recommendations in the Guide for the Care and Use of Laboratory Animals of the National Institutes of Health. The protocol was approved by the Institutional Animal Care and Use Committee of Northern Jiangsu Province Hospital, Clinical Medical College, Institute of General Surgery - Yangzhou, Yangzhou University.

### Study subjects

The gastric cancer tissues and adjacent normal tissues (5 cm above cancerous parts and without cancer tissues as verified by a pathologist) were collected from 65 patients with primary gastric cancer who had undergone surgical resection in Northern Jiangsu Province Hospital, Clinical Medical College, Institute of General Surgery - Yangzhou, Yangzhou University from February 1, 2015 to February 1, 2017. All tissues were collected from 42 males and 23 females ranging from 29 to 82 years old, with the mean ages of (57.35 ± 17.74) years. All enrolled patients were confirmed to have primary gastric cancer, among which, 20 cases were diagnosed as non-regional lymph node metastasis (LNM) (N0), 13 cases with 1 - 6 regional LNM (N1), 19 cases with 6 - 15 regional LNM (N2) and 13 cases with over 15 regional LNM (N3). None of the enrolled patients had received any chemotherapy or radiotherapy prior to surgery. The patients with gastric remnant carcinoma who received gastric surgery or had severe cardiopulmonary dysfunction complications were excluded. Part of the collected tissues was immediately stored in liquid nitrogen, while the remaining tissues were fixed by paraformaldehyde and embedded in paraffin for subsequent experiments.

### Cell culture

Gastric cancer cell lines (BGC-823, SGC7901, MKN45, MKN28, AGS, and HGC-27) and normal gastric mucosal epithelial cell line GES-1 were cultured in Roswell Park Memorial Institute (RPMI)-1640 medium containing 10% fetal bovine serum (FBS), 100 U/mL penicillin and streptomycin solution. The AGS cell line was cultured in F12 medium supplemented with 10% FBS, 100 U/mL penicillin and streptomycin solution. All cells were incubated at 37°C with 5% CO_2_. The above cell lines were purchased from Procell Life Science and Technology Co., Ltd. (Wuhan, China) (http://www.procell.com.cn/).

### Cell treatment

The selected gastric cancer cell line SGC7901 was transfected with siRNA targeting lncRNA XIST-1 (si-XIST-1) and XIST-2, miR-132 mimic, miR-132 inhibitor, PXN overexpression plasmid (oe-PXN), co-transfected with miR-132 mimic and si-XIST, and co-transfected oe-PXN and si-XIST or their negative control (NC) plasmids such as si-NC, mimic-NC, inhibitor-NC and oe-NC. Si-XIST, miR-132 mimic, miR-132 inhibitor and oe-PXN plasmids were all purchased from Guangzhou RiboBio Co., Ltd. (Guangdong, China).

When cell confluence reached 50% - 60%, the gastric cancer cells were seeded into a 24-well plate and transfected according to Lipofectamine^TM^ protocols (Invitrogen Inc., Carlsbad, CA, USA). Lipofectamine 2000 (1 μL lipofectamine 2000 + 50 μL serum-free medium placed at room temperature for 5 min) and RNA ready for transfection (20 pmoL RNA ready for transfection + 50 μL serum-free medium) were mixed. The mixture was then added to the cells for transfection, followed by incubation with culture medium at 37°C and with 5% CO_2._

### Fluorescent in situ hybridization (FISH)

FISH kit (C10910, Guangzhou RiboBio Co., Ltd., Guangdong, China) was used for in situ detection of lncRNA XIST expression in gastric cancer cells. After the cover glasses were placed at the bottom of a 24-well plate, the cells in logarithmic growth phase were detached onto the glasses (about 6 × 104 cells/well), and then fixed with 4% paraformaldehyde at room temperature for 10 min. Subsequently, the cells in each well were added with 1 mL pre-cooled permeable liquid and allowed to stand at 4°C for 5 min, and the permeable liquid was removed. Next, the cells in each well were added with 200 μL pre-hybridization solution and sealed at 37°C for 30 min. Following that, 2.5 μL of 20 μM FISH Probe Mix stock solution was added into hybridization solution by avoiding exposure to light, with pre-hybridization solution in each well discarded. Then, the cells were hybridized with probe hybridization solution overnight at 37°C, followed by washing with lotion I at 42°C to reduce background signal, then washed with lotion II and lotion III at 42°C, and lastly rinsed with 1 × PBS. The above procedures were all conducted by avoiding exposure to light. Afterwards, the cells were stained with 4',6-diamidino-2-phenylindole (DAPI) dye for 10 min in the dark. The cover glasses were carefully taken out from each well and fixed on a glass slide using mounting medium in the dark, for the fluorescence detection. The specific probes of lncRNA XIST were synthesized by Guangzhou RiboBio Co., Ltd. (Guangdong, China).

### Dual-luciferase reporter gene assay

The biological prediction website was used to analyze the putative binding sites between lncRNA XIST, miR-132 and PXN, as well as to obtain the fragment sequence containing the active site in the gene. Full length lncRNA XIST and the 3’untranslated region (UTR) of PXN were separately amplified and cloned into pmirGLO (E1330, Promega Corporation, Madison, WI, USA) luciferase vector, namely plncRNA XIST-wild type (WT) and pPXN-WT. Next, the plncRNA XIST-mutant type (MUT) and pPXN-MUT vectors were constructed, with renilla luciferase-expressed pRL-TK vector (E2241, Promega Corporation, Madison, WI, USA) as an internal reference. The miR-132 mimic and mimic-NC were then separately co-transfected into SGC7901 cells (CRL-1415, American Type Culture Collection Company, Manassas, VA, USA) with recombinant luciferase reporter vectors. Lastly, Dual Luciferase Reporter Gene Assay Kit (GM-040502A, Shanghai Qian Chen Bio Science and Technologies Co., Ltd., Shanghai, China) was utilized for the luminance detection at 560 nm [firefly relative light unit (RLU)] and 465 nm (renilla RLU). The luciferase activity was expressed by the ratio of firefly RLU to renilla RLU.

### RNA pull-down assay

Cell lysates were prepared using RNA immunoprecipitation (RIP) solution and then equally allocated into several tubes (one tube used as input) and stored at -80°C for subsequent experiments. According to the instructions of the Magnetic RNA-protein Pull-down Kit (Pierce Biotechnology Inc, Rockford, IL, USA), 1 μg of biotin-labeled RNA was added with 500 μL of structure buffer, water bathed at 95°C for 2 min and then ice bathed for 3 min. When the full resuspension of the magnetic beads was observed, the EP tube was added with 50 μL of magnetic bead suspension, incubated at 4°C overnight and subsequently centrifuged at 1610 g for 3 min with the removal of the supernatant. Later, the suspension was washed with 500 μL RIP wash buffer for 3 times, added with 10 μL of cell lysis buffer and allowed to stand at room temperature for 1 h. Lastly, the incubated proteins in the magnetic RNA-protein mixture were eluted, and the protein concentration was detected by bicinchoninic acid (BCA) assay and protein expression determined by western blot analysis.

### RNA immunoprecipitate (RIP) assay

Cells were lysed using lysis buffer [25 mM Tris-HCl pH 7.4, 150 mM NaCl, 0.5% NP-40, 2 mM Ethylene Diamine Tetraacetic Acid (EDTA), 1 mM NaF and 0.5 mM dithiothreitol] containing RNasin (Takara Holdings Inc., Kyoto, Japan) and protease inhibitor mixture (B14001a, Hoffmann-La Roche Ltd, Basel, Switzerland). After centrifugation at 12000 × g for 30 min, magnetic beads coated with antibody anti-human Ago-2 (BMFA-1, Biomarker Technologies Co., Ltd., Beijing, China) were added to the lysate, while the control group was added with magnetic beads coated with the antibody to immunoglobulin G (IgG). After that, the beads were incubated at 4°C for 4 h and washed with washing buffer (50 mM Tris-HCL, 300 mM NaCl pH 7.4, 1 mM MgCl2, and 0.1% NP-40) for 3 times. Lastly, Trizol was used to extract RNA from the beads, followed by detection of lncRNA XIST by RT-qPCR.

### RT-qPCR

The gastric cell line SGC7901 in the logarithmic growth phase was collected for transfection. The total RNA of the cells was extracted using TRIzol (15596026, Invitrogen, Car, Cal, USA) after 24-h transfection. Next, RNA was reversely transcribed into complementary DNA (cDNA) according to the instructions of PrimeScript RT reagent kit (RR047A, TaKaRa, Tokyo, Japan). Primers of lncRNA XIST, miR-132, PXN, U6 and glyceraldehyde-3-phosphate dehydrogenase (GAPDH) were designed and synthesized by Shanghai Sangon Biological Co., Ltd. (Shanghai, China) (Table 1). Then, in accordance with the instructions of EasyScript First-Strand cDNA Synthesis SuperMix (AE301-02, TransGen Biotech Co., Ltd., Beijing, China), 20 μL of reverse transcription system was applied. Then, real time qPCR was conducted using the ABI7500 fluorescence quantitative PCR of ABI Company (Oyster Bay, NY, USA). 2^-ΔΔCt^ represents the ratio of target gene expression in the experimental group to the control group.

**Table 1:** Primer sequences for RT-qPCR.

**Genes**	**Sequences (5’-3’)**
lncRNA XIST	F: CTCTCCATTGGGTTCAC
	R: GCGGCAGGTCTTAAGAGATGAG
miR-132	F: TGGATCCCCCCCAGTCCCCGTCCCTCAG
	R: TGAATTCGGATACCTTGGCCGGGAGGAC
PXN	F: TGAAACTGGTTGAAGGGTGT
	R: GACACCAGCTTTCCTGAGAA
GADPH	F: GCACCGTCAAGGCTGAGAAC
	R: TGGTGAAGACGCCAGTGGA
U6	F: TGCGGGTGCTCGCTTCGGCAGC
	R:CCAGTGCAGGGTCCGAGGT

RT-qPCR, reverse transcription quantitative polymerase chain reaction; F, forward; R, reverse; U6, Small nuclear ribonucleic acid 6; GAPDH, glyceraldehyde-3-phosphate dehydrogenase; LncRNA, long non-coding RNA; miR-132, microRNA-132; PXN, Paxillin.

### Western blot analysis

SGC7901 cells after 48 h of transfection were washed with pre-cooled PBS, lysed on ice with prepared radio-Immunoprecipitation assay (RIPA) lysis buffer for 30 min and centrifuged at 14000 ×g with supernatant collected. After protein concentration was determined by the BCA method, cells were stored at -20°C for subsequent experiments. Following that, sodium dodecyl sulfate polyacrylamide gel electrophoresis (SDS-PAGE) was performed to isolate proteins which were subsequently wet-transferred onto a nitrocellulose membrane, and sealed with 5% bovine serum albumin (BSA) at room temperature for 1 h. Subsequently, the membrane was added with diluted primary antibody to PXN (ab32084, 1 : 1000) overnight at 4°C. Then, the membrane was washed with phosphate buffer saline-Tween 20 (PBST) for 3 times (10 min each), followed by incubation with secondary antibody to IgG (ab205718, 1 : 2000) diluted with 5% skim milk, and placed on an oscillator table at room temperature for 1 h. The membrane was then washed with PBST again for 3 times (15 min each) and developed with developer using Bio-Rad Gel Imaging System (MG8600, Beijing Thmorgan Biotechnology Co., Ltd., Beijing, China). IPP7.0 software (Media Cybernetics, Singapore) was applied for quantitative analysis. The ratio of gray value of PXN band to internal control GAPDH referred to their respective levels. All the aforementioned antibodies were purchased from Abcam Company (Cambridge, UK).

### 5-Ethynyl-2’-deoxyuridine (EdU) assay

EdU detection kit was purchased from RiboBio Co., Ltd. (Guangdong, China) and Triton X was purchased from Beijing Solarbio Life Sciences Co., Ltd. (Beijing, China). Cells in exponential growth phase were seeded into a 96-well plate (5 × 10^4^ cells/well). When cells were adherent to the wall, cells in each well were added with 500 μL of 50 μmol/L EdU medium, incubated at 37°C for 2 h, fixed with 40 g/L paraformaldehyde for 20 min, incubated with 2 mg/mL glycine for 10 min and washed twice with PBS. After that, the cells were permeabilized using 500 μL 0.5% Triton X, cultured with Apollo dye reaction fluid at room temperature for 30 min in the dark, incubated with Hoechst 33342 reaction fluid at room temperature void of light for 30 min, and washed twice with 0.5% Triton X. Lastly, the cells were observed under an inverted fluorescent microscope and counted by Image-Pro Plus 6.0 (IPP).

### Scratch test

A straight line on the cell surface was made using a 200 μL sterile micropipette, followed by 3 PBS washes. Then, the cells were photographed under an inverted microscope (CX23, Olympus Optical Co., Ltd., Tokyo, Japan) (× 100). After 48 h of incubation, the 6-well plate was taken out again and cells were photographed to measure wound healing rate.

### Transwell assay

Matrigel (Becton, Dickinson and Company, NJ, USA) was diluted with pre-cooled serum-free Dulbecco’s modified eagle’s medium (DMEM) (1 : 100). Later, the solution was completely mixed and added into apical Transwell chambers (100 μL each). The chambers were incubated at room temperature for 2 h and washed with 200 μL of serum-free RPMI 1640 medium. After 24 h of transfection, cells were detached, resuspended with serum-free DMEM, counted, and diluted at a concentration of 3 × 10^5^ cells/mL. Then, 100 μL diluted cell suspension was added to the Transwell apical chamber (Corning Glass Works, Corning, N.Y., USA), while the basolateral chamber was supplemented with 600 μL DMEM medium containing 10% serum (chemotactic factor) following the instructions of Transwell Chamber Kit. Lastly, cells were stained by crystal violet and 3 fields were randomly selected for counting the number of cells crossing membrane.

### Flow cytometry

Annexin V-fluorescein Isothiocyanate/Propidium Iodide (FITC/PI) Staining Kit (556547, Shanghai Shuojia Biotechnology co., Ltd., Shanghai, China) was used to measure the cell apoptosis of SGC7901 after 48-h transfection. Deionized water was used to dilute 10 × binding buffer into 1 × binding buffer. After centrifugation at 715 × g for 5 min, cells were collected, resuspended with pre-cooled 1 × PBS, and centrifuged again at 7 ×g for 5 - 10 min. Cells were then resuspended in 300 μL 1 × binding buffer, mixed with 5 μL Annexin V-FITC, and incubated at room temperature avoiding exposure to light for 15 min. Subsequently, cells were added with 5 μL PI for 5 min for detection on a flow cytometer (Cube6, Partec, Germany) and ice-bathed for 5 min in the dark. FITC signal was detected at an excitation wavelength of 480 nm and 530 nm, while PI signal was detected at an excitation wavelength over 575 nm.

### Tumor xenograft in nude mice

A total of 66 BALB/c nude mice (aged 4 weeks, weighing 18 - 25 g, irrespective of gender) were purchased from Shanghai SLAC Laboratory Animal Co., Ltd. (Shanghai, China) and fed under specific pathogen-free (SPF) environment (5 mice per group). A total of 1 × 10^6^ SGC7901 cells were subcutaneously inoculated into nude mice, the tumor volume was monitored once a week and calculated using V = π/6 (height × length × width). The nude mice were euthanized at the end of the third week. The tumors were collected and the weight of the tumors was measured.

### Statistical analysis

All data were analyzed using SPSS 21.0 software (IBM Corp. Armonk, NY, USA). The measurement data were presented as the mean ± standard deviation. If the data conformed to normal distribution and homogeneity of variance, comparisons between two groups were analyzed by *t*-test, while comparisons among multiple groups were analyzed using one-way analysis of variance (ANOVA) with Tukey’s post-hoc test. When the data were in skew distribution and heterogeneity of variance, the non-parametric rank sum test was performed. A value of p < 0.05 was considered as statistically significant.
